The article "Optimization of Personnel Placement Scheme and Big Data Analysis Based on Multilayer Variable Neural Network Algorithm" was retracted in 2023. Reasons: suspected computer-generated content; unreliable results or conclusions; concerns about the data; concerns about the results or conclusions.

# Optimization of Personnel Placement Scheme and Big Data Analysis Based on Multilayer Variable Neural Network Algorithm

**DOI:** 10.1155/2021/3250062

**Published:** 2021-10-18

**Authors:** Haiqiu Li

**Affiliations:** Department of Business Administration, Zhejiang Technical Institute of Economics, Hangzhou 310016, China

## Abstract

People usually use the method of job analysis to understand the requirements of each job in terms of personnel characteristics, at the same time use the method of psychological measurement to understand the psychological characteristics of each person, and then put the personnel in the appropriate position by matching them with each other. With the development of the information age, massive and complex data are produced. How to accurately extract the effective data needed by the industry from the big data is a very arduous task. In reality, personnel data are influenced by many factors, and the time series formed by it is more accidental and random and often has multilevel and multiscale characteristics. How to use a certain algorithm or data processing technology to effectively dig out the rules contained in the personnel information data and explore the personnel placement scheme has become an important issue. In this paper, a multilayer variable neural network model for complex big data feature learning is established to optimize the staffing scheme. At the same time, the learning model is extended from vector space to tensor space. The parameters of neural network are inversed by high-order backpropagation algorithm facing tensor space. Compared with the traditional multilayer neural network calculation model based on tensor space, the multimodal neural network calculation model can learn the characteristics of complex data quickly and accurately and has obvious advantages.

## 1. Introduction

People usually use the method of job analysis to understand the requirements of each job position in terms of personnel characteristics, use the method of psychological measurement to understand the psychological characteristics of each personnel member, and then place the personnel in the appropriate position through mutual matching [1–3]. It is often difficult for people to understand the massive data stored, and they cannot draw accurate and effective conclusions from these data, because people lack effective methods and practical technologies to extract valuable information from massive data. How to use a certain algorithm or data processing technology to effectively mine the laws contained in personnel information data and explore personnel placement scheme has become an important topic [4, 5]. Big data has the characteristics of large quantity, many types, fast speed, and difficult discrimination. The rapid development of video media, social network, Internet of things, and other industries poses a severe challenge to the rapid and accurate processing of big data [6, 7]. With the rapid development of Internet technology and the era of big data, artificial neural network (ANN) has become one of the most popular algorithms in modern times [8]. In recent years, neural network algorithms have made great progress in both theoretical research and practical application. More and more neural networks with different structures have been proposed and applied to more and more complex artificial intelligence tasks [9–11]. The mixed reform of state-owned enterprises may involve changing the original ownership structure of the enterprise or changing the original labor employment and distribution incentive system. This series of reforms is related to the vital interests of employees [12]. In order to ensure the success and steady promotion of this reform, we should pay special attention to the placement of employees. The current datasets show little change due to their specific composition; that is, each of them consists of only a single scene or domain [13]. Therefore, the models trained on these datasets are not robust enough. At present, deep learning has become an important research direction in the field of artificial intelligence because it can imitate the structure of human brain, extract and abstract information, and solve problems in real life [14–16]. Deep learning is a mathematical model composed of several neurons connected with each other to process complex information, which can reduce human workload and enhance the accuracy of actual results. Convolutional neural network is easy to fall into local optimal solution when using gradient descent algorithm to train parameters in forward propagation. At the same time, gradient dispersion is easy to occur with the increase of layers in the process of back propagation [17]. BP (backpropagation) algorithm of multilayer convolutional neural network calculates the weight and threshold of neural network based on neural learning rules [18]. This algorithm can converge when the step size of the network weight and threshold is adjusted infinitely every time, and the introduction of momentum factor can speed up the calculation [19].

With the continuous development of artificial intelligence technology and human resources market, a large amount of personnel data with rich information has been produced. Rich but difficult to use data resources have become a common phenomenon in today's society, which has become an obstacle for people to using information efficiently [20]. In order to place people with different characteristics in their suitable jobs, the constraint satisfaction model of artificial neural network is used to solve this problem. Each node in the model represents a hypothesis, and the connection weight of each node represents the constraints between the hypotheses. At the same time, each node can have input from the outside world, and a certain bias value can be set for the network when necessary [21]. With the development of the network, the amount of network data increases gradually, and the structure of the network becomes more and more complex, which will lead to a larger amount of network parameters. In the face of massive network parameters, this leads to network training and testing, which has high requirements for GPU memory and computing power [22]. In reality, personnel data is affected by many factors, and the time series formed by it has greater contingency and randomness and often has multilevel and multiscale characteristics. The single neural network prediction model has limitations, which has a certain impact on the prediction accuracy of personnel placement data [23]. Based on the traditional data processing of multilayer variable neural network, this paper captures the distribution characteristics of data in high-order tensor space, establishes a multimodal neural network calculation model for complex big data feature learning, and realizes the optimization of personnel placement scheme.

## 2. Related Work

With the continuous development of the Internet and the human resources market, a large amount of personnel data with rich information has been produced. With the popularization of big data technology, it is possible to deal with massive personnel data. Literature [24] suggested that the production of labor force is the production of human life and consumption. The total population and population composition, consumption level, and consumption structure in society directly determine the supply of labor force. Literature [25] showed that the level of production development, the scale and speed of economic growth, and the reasonable coordination degree of economic structure determine the status of jobs that the society can provide, thus determining the demand for labor. Literature [26] holds that the supply and demand of labor force are in unity of opposites, which not only restricts but also affects the production and reproduction of labor force itself. Literature [27] pointed out that when the supply and demand of labor force are balanced, the full employment of the working people has a realistic possibility, and they can complete the process of “labor force to wage,” thus ensuring the production and reproduction of labor force. Literature [28] holds that there is an inverse relationship between unemployment rate and wage growth rate, or between unemployment rate and inflation rate, which is also a theoretical basis for western market economy countries to govern unemployment and inflation. Literature [29] studied the stochastic optimization method of cluster analysis to select stocks for investment. The traditional analysis method is simple and easy to master, but the change of personnel placement data often presents nonlinear characteristics, and the traditional prediction method is based on linear change modeling, so the accuracy of the analysis and prediction of personnel placement data is low.

The multimodal neural network calculation model simultaneously extends the learning model from the vector space to the tensor space. Through the high-order back propagation algorithm oriented to the tensor space, the parameters of the neural network are reversed. The multimodal neural network calculation model can quickly and accurately learn the characteristics of complex data, which has obvious advantages over the conventional multilayer neural network calculation model based on tensor space. From the perspective of laborers, under the new employment policy, they must bear certain risks and pressures, and at the same time, they will enjoy development prospects and hopes they have never had in the past, i.e., the prospects and hopes of getting the fullest use and realization, so that they can make their own talents. The social placement of human resources can reduce or eliminate employment insecurity, but in terms of individuals, they lose the freedom to choose a career.

## 3. Methodology

### 3.1. Multilayer Neural Network

Multilayer neural network learning can be regarded as a nonlinear system *T* with *n* layers, *T*=(*T*1, *T*2,…, *Tn*), I and O represent the input data and output of the system, respectively. The neural network structure is shown in Figure 1.

After the data has undergone the n-layer system transformation, the input and output data are still equal, which means that after the data passes through the n-layer system, the input and output of each layer are equal, and no effective information is lost. In the training process of the big data multilayer neural network model, the learning of its parameters and structure should be autonomous, that is, without human intervention, so that the multilayer neural network learning model can autonomously learn the multilayer features of the data.

According to the characteristics of the input layer, the latitude of neurons in the input layer is mainly determined according to the different attributes and types of samples, and the input layer should fully consider the latitude of all data and the accuracy of related attributes [30–32]. From the characteristics of hidden layer, hidden layer is mainly composed of data thresholds and related conditions provided by users. As an important limiting condition, hidden layer can change the activity of neurons and ensure the flexibility and variability of prediction model. Each neuron has an input and an output. The input and output of the input layer are the attribute values of training samples. The training of multilayer neural network learning model includes two steps: first training and retraining. In the first training stage, the established model neural network is trained layer by layer from bottom to top to obtain initial parameters. In the retraining stage, the existing data is used to correct the parameters once from top to bottom, so as to obtain the final correct parameters.

The operation process mainly includes three stages: convolution, nonlinear transformation, and downsampling. As the main component of the network, the convolutional layer not only undertakes most of the network calculations, but also is a key step in feature extraction. The convolutional layer extracts effective feature values through a specific convolution kernel and a convolution operation on the input picture. After multiple convolution operations, the part of the feature that matches the features of the convolution kernel is strengthened, so that the parameters after training can extract the best data features. In the convolution stage, the features of the original input signal are extracted to determine the number of convolution kernels, and the convolution kernels with key features of the original signal can realize weight sharing. The first-stage convolution formula is shown in the following equation:

(1) $$\begin{array}{c} y_{i}=b_{j}\sum_{i}w_{ij}x_{i}. \end{array}$$

Among them, *x*_*i*_ is the input of the multilayer neural network, which is composed of *n* two-dimensional data, and *y*_*i*_ is the output of the multilayer neural network and is composed of *m* two-dimensional data; and *b*_*j*_ is the bias vector. In the nonlinear transformation stage, the output needs to be nonlinearly activated, and the most used activation function is the Sigmoid function:

(2) $$\begin{array}{c} f\left(y\right)=\frac{1}{\left(1+e^{-y}\right)}. \end{array}$$

In the downsampling stage, the processing of features usually adopts a pooling method. The pooling operation allows the data to maintain most characteristics while greatly reducing the amount of data. By using W weights to connect convolutional neurons, a deep learning model based on multilayer networks can be constructed.

Average pooling algorithm is as follows:

(3) $$\begin{array}{c} x_{j}^{l}=do\;wn\left(x_{j}^{l-1}\right). \end{array}$$

Maximum pooling algorithm is as follows:

(4) $$\begin{array}{c} x_{j}^{l}=f\left(\beta_{j}^{l}do\;wn\left(x_{j}^{l-1}\right)+b_{j}^{i}\right), \end{array}$$

where down(*x*_*j*_^*l*−1^) represents the downsampling operation, which can perform dimensionality reduction operations on the data by block.

The training methods of multilayer neural network mainly include pretraining and fine-tuning. The pretraining mainly adopts back propagation and gradient descent algorithm, which is an unsupervised training process. After the pretraining, the parameters are fine-tuned through supervised training. The output of a typical single-depth model of neural network is shown in Figure 2.

Multilayer neural network has different optimization strategies, and there are many differences in applicable problems and information processing methods. Multilayer neural network can be used for pattern recognition, optimal control, and load forecasting.

### 3.2. Constraint Satisfaction Model

The constraint satisfaction model established in this paper is a model in multilayer neural network [33–35]. Each node in the model represents a hypothesis. The model consists of a set of variables and a set of constraints. A given set of constraints is satisfied by assigning values to a set of variables. For each node, there can be input from the outside, which reflects external evidence. When necessary, a certain bias value can be set for the network to reflect the predisposition of the decision maker. These can be regarded as various constraints. Their constraint strength can be expressed by the value of *w*, input, and bias. The degree to which the final decision (i.e., personnel placement) satisfies these constraints can be measured by goodness. The fitness goodness_*i*_ for a certain node *i* can be calculated by the following formula:

(5) $$\begin{array}{c} {\text{goodness}}_{i}=\sum_{j}w_{ij}a_{i}a_{j}+{\text{bias}}_{i}a_{i}+{\text{input}}_{i}a_{i}. \end{array}$$

In the formula, *a*_*i*_ is the activation value of the receiving node *i*, *a*_*j*_ is the activation value of the sending node *j*, and *w*_*ij*_ is the connection weight between them. *bias*_*i*_ is the bias value of node *i*, and input_*i*_ is the external input of node *i*. The fitness of the entire network is the sum of the fitness of all receiving nodes in the network, expressed by the following formula:

(6) $$\begin{array}{c} \text{goodness}=\sum_{ij}w_{ij}a_{i}a_{j}+\sum_{i}{\text{bias}}_{i}a_{i}+\sum_{i}{\text{input}}_{i}a_{i}. \end{array}$$

The network maximizes goodness by constantly updating the activation value of each node. It can be seen from formula (5) that the goodness_*i*_ of node *i* is related to the input from other nodes, the outside world, and the prebias value, which can be regarded as the input value *net*_*i*_ of node *i*, which is defined as

(7) $$\begin{array}{c} {\text{net}}_{i}=\mathrm{int}\left(\sum_{j}w_{ij}a_{i}a_{j}+{\text{bias}}_{i}\right)+ext\left({\text{input}}_{i}\right), \end{array}$$

where (∑_*j*_*w*_*ij*_*a*_*i*_*a*_*j*_+bias_*i*_) represents the input of node *i* from the inside of the network, and input_*i*_ represents the input of node *i* from the outside of the network. The coefficients *int* and *ext*, respectively, reflect the relative degree of influence of the input from the inside and from the outside on the node *i*. If *int* is greater than *ext*, the amount of input received from the inside will have a greater impact, and vice versa. If the *net*_*i*_ obtained according to equation (3) is positive, then the node will update its activation value as follows:

(8) $$\begin{array}{c} a_{i}\left(t+1\right)=a_{i}\left(t\right)+{\text{net}}_{i}\left[\text{ceiling}-a_{i}\left(t\right)\right]. \end{array}$$

In the formula, *a*_*i*_(*t*+1) is the activation value after the update, *a*_*i*_(*t*) is the activation value before the update, and ceiling is the maximum activation value that all nodes can reach. If *net*_*i*_ is negative, then the node will update the activation value as follows:

(9) $$\begin{array}{c} a_{i}\left(t+1\right)=a_{i}\left(t\right)+{\text{net}}_{i}\left[a_{i}\left(t\right)-\text{floor}\right], \end{array}$$

where floor is the minimum activation value of all nodes. By using formulas (8) and (9), the goodness of the whole network will gradually increase and finally reach an extreme value. This means that, in this state, various constraints of the network have been met to the greatest extent. The optimal step size can be obtained when the optimization calculation is carried out along the negative gradient direction, and the search directions of adjacent two times are orthogonal. When the gradient optimization method is far away from the minimum point, the function value decreases more and converges faster. When approaching the minimum point, the sawtooth phenomenon is formed, the traveling distance is shortened, and the convergence speed is slowed down.

## 4. Result Analysis and Discussion

### 4.1. Data Processing

We selected the employment data from May 1, 2016, to May 1, 2020, as training samples and the employment data from May 1, 2019, to May 1, 2020, as model forecast data. The selected data is very big, 5 years, and it can be called big data [36–44]. The fluctuation of the personnel placement is shown in Figure 3.

When a given training sample is used to train the network, choosing an appropriate optimization algorithm to optimize the network weights is the most critical step affecting the network training effect. The performance of the optimization algorithm not only affects the final effect of network training, but also affects the time and other resources consumed in the training process. Because the fluctuation of personnel placement data with time is characterized by high noise and nonlinearity, wavelet analysis can be used for multiresolution analysis, and the signals can be observed gradually from coarse to fine. Using wavelet analysis, the data curve of personnel placement is decomposed into two parts: low frequency and high frequency. According to Mallat algorithm, db5 wavelet is selected as the basis function to decompose the original data with four layers of wavelet. The result after wavelet analysis is shown in Figure 4. Among them, d1 wavelet is the low-frequency part, and d2, d3, and d4 wavelets are the high-frequency part.

It can be seen from Figure 4 that the low-frequency wavelet and the original wavelet have basically the same change trend, and the high-frequency wavelet fluctuates up and down around zero value, which proves that the original wavelet decomposition has achieved good results. Because the mapping relationship between input and output of neural network can be linear or nonlinear, multilayer neural network does not use certain mathematical functions to express its inherent rules. In the process of network training, by inputting a large number of learning samples, the network can learn this specific mapping ability. Multilayer neural network belongs to supervised learning, which needs label signal to guide learning. After the samples are input into the multilayer neural network, an output signal will be obtained through the complex internal mapping relationship. The optimizer compares the output signal and the label of the samples to update the weights of each neuron, and the judgment standard of this difference is judged by the loss function. The smaller the loss function value, the better the training effect. The function of the optimizer is to find the optimal weight of the network, so that the loss function is as small as possible.

### 4.2. Model Prediction

Because the numerical range of personnel placement data is not large, in order to ensure the accuracy of prediction results, neural network is not normalized before training. Low-frequency wavelet represents the long-term trend of personnel placement data, and multilayer variable neural network with memory function is used for training. High-frequency wavelet is the performance of personnel placement data affected by accidental factors, which has strong randomness. Therefore, multilayer variable neural network with good approximation to nonlinear function is used for training. In Elman neural network, tansig function is used in the hidden layer, purelin function is used in the output layer, and trainlm is used as the learning function. In multilayer variable neural network, tansig function is used as hidden layer, and traingdm is used as learning function.

MATLAB is used for simulation, and then according to the reconstruction formula, the coefficients of each layer of the predicted wavelet are reconstructed, and the reconstructed wavelet with the same time scale as the original wavelet is obtained, that is, the wave curve of personnel placement optimization. The result of comparing the predicted values obtained by neural network training with the actual values is shown in Figure 5.

Due to facing specific problems, it is necessary to design different loss functions and activation functions. Loss function is an index reflecting the fitting degree of multilayer variable neural network and training data. The worse the fitting degree is, the greater the value of loss function should be. Because the traditional optimization algorithm needs to optimize according to the gradient of the function, when the loss function is relatively large, its corresponding gradient can be large enough, so that the update speed is fast enough. There are two main points in choosing a suitable loss function: firstly, it can reflect the true label of solving the problem; secondly, the loss function should have a reasonable gradient, which is conducive to solving the gradient, and then the weights and parameters can be updated. By comparing the actual values, general neural network prediction results, and multilayer variable neural network prediction results, as shown in Figure 6, it can be seen that the accuracy of multilayer variable neural network in predicting personnel placement is higher than that of nonoptimized neural network.

The neural network model is used to train the sample data. The number of hidden layer units is determined to be 30 by trial and error method. The maximum training times max_epoch = 600, and the target error err_goal = 1 × 10^−6^ are set. By comparison, it can be seen that the difference between the predicted value and the actual value is small, and the trend of the two values is basically the same. The predicted value changes slightly earlier than the actual value, which can achieve the actual effect of prediction. The MSE of neural network is calculated to be 6.5488 × 10^−6^.

From the prediction data, the neural network model has better prediction performance, smaller relative error, and more accuracy. Through the research and implementation of the prediction of personnel placement based on big data and multilayer variable neural network, it can be found that the model can combine the advantages of big data and neural network and has a very good prediction effect on personnel placement. Therefore, it is of great significance to predict the personnel placement based on big data and multilayer variable neural network.

## 5. Conclusions

Data mining technology can automatically extract the internal relations of economic activities from historical data, overcome many limitations and difficulties faced by traditional quantitative forecasting methods, and avoid the influence of many human factors. Big data has the characteristics of high complexity, real-time variability, and so on. Because of its extensive sources and diverse types, big data will contain a variety of complex combination types. At the same time, the system is required to be able to process different data of new buildings in real time. Multilayer variable neural network effectively solves the problem of nonadaptive static learning model and has obvious advantages in dealing with the complexity and real-time variability of big data. This study suggests that the constraint satisfaction model can be used for personnel placement, and the simulation experiment also proves the feasibility of this method. This model provides a way to forecast employment based on massive personnel data. In this model, the wave curve of personnel placement data is decomposed into different layers of data with different frequencies by wavelet decomposition, and the prediction results are reconstructed by wavelet transform using multilayer neural network. The model is used to study and predict the data of personnel placement, and the results show that the combined model has high accuracy. Multilayer neural network learning model can deal with a large amount of data accurately and carry out complex training, which will also take more time correspondingly. In order to improve the training speed of multilayer neural network learning model, the best way is to make full use of cloud computing technology to optimize the neural network computing model.

The problem of difficult resettlement of unemployed people is mainly due to the economic structure, which cannot be solved in a short time. To promote employment, we should not solely rely on the speed of economic growth and investment in fixed assets, but also explore new ways to find an economic development mode that is conducive to expanding employment. It is necessary to communicate with employees many times to form diversified resettlement channels, which are chosen by employees independently, so as to ensure legal compliance and win-win situation for all parties.

## Figures and Tables

**Figure 1:** Multilayer neural network learning model.

**Figure 2:** Multilayer network single-depth model output results.

**Figure 3:** Fluctuations of original personnel placement data.

**Figure 4:** Data diagram of different bands after wavelet decomposition.

**Figure 5:** Comparison of actual and predicted values of personnel placement data.

**Figure 6:** Comparison of multilayer variable neural network with general neural network and actual values.

## Data Availability

The data used to support the findings of this study are available from the corresponding author upon request.

## References

[1] Talasila V., Madhubabu K., Madhubabu K., Mahadasyam M., Atchala N., Kande L. (2020). The prediction of diseases using rough set theory with recurrent neural network in big data analytics. *International Journal of Intelligent Engineering and Systems*.

[2] Yeh L.-Y., Tsaur W.-J., Huang H.-H. (2017). Secure IoT-based, incentive-aware emergency personnel dispatching scheme with weighted fine-grained access control. *ACM Transactions on Intelligent Systems and Technology*.

[3] Maitrey P. S. (2020). A dual security scheme based on DWT for personnel authentication. *International Journal of Engineering and Advanced Technology*.

[4] Onan A. (2020). Sentiment analysis on product reviews based on weighted word embeddings and deep neural networks. *Concurrency and Computation: Practice and Experience*.

[5] Tien Bui D., Nhu V.-H., Hoang N.-D. (2018). Prediction of soil compression coefficient for urban housing project using novel integration machine learning approach of swarm intelligence and multi-layer perceptron neural network. *Advanced Engineering Informatics*.

[6] Orujov F., Maskeliūnas R., Damaševičius R., Wei W. (2020). Fuzzy based image edge detection algorithm for blood vessel detection in retinal images. *Applied Soft Computing*.

[7] Onan A., Tocoglu M. A. (2021). A term weighted neural language model and stacked bidirectional LSTM based framework for sarcasm identification. *IEEE Access*.

[8] Adhikari S. P., Yang C., Slot K., Strzelecki M., Kim H. (2018). Hybrid no-propagation learning for multilayer neural networks. *Neurocomputing*.

[9] Ding M., Gao Y., Chen X. (2017). Multi-layer neural network stock prediction model based on the background of big data. *Software*.

[10] Vinichenko M. V., Karácsony P., Kirillov A. V. (2017). Increase of efficiency of stimulation of a personnel reserve of the educational organization. *Man in India*.

[11] Li S., Zhao Y., Fan K., Zhang Y. (2020). Application of neural network in structural damage diagnosis. *Journal of Building Science and Engineering*.

[12] Ge J., Zhao W., Xu Y. (2020). Research on DDoS attack detection method of big data cloud platform based on neural network. *Modern Electronic Technology*.

[13] Peng D., Lan M., Li S. (2018). Modeling research on boiler combustion oxygen content based on big data and neural network. *Thermal Energy and Power Engineering*.

[14] Huang H., Yu H. (2018). A layerwise tensorized compression of multilayer neural network. *IEEE Transactions on Neural Networks and Learning Systems*.

[16] Salih Ageed Z., Zeebaree R. M., Mohammed Sadeeq M. (2021). Comprehensive survey of big data mining approaches in cloud systems. *Qubahan Academic Journal*.

[17] Jiang L. (2018). Analysis on how to strengthen the management of military personnel placement files under the background of big data. *Shandong Archives*.

[18] Cui H. (2020). The construction of digital expropriation and resettlement system based on GIS. *China New Technology & New Products*.

[19] Ramakrishnan V., Ramesh K. (2017). Scanning schemes in white light photoelasticity - Part II: novel fringe resolution guided scanning scheme. *Optics and Lasers in Engineering*.

[20] Höpken W., Eberle T., Fuchs M. (2021). Improving tourist arrival prediction: a big data and artificial neural network approach. *Journal of Travel Research*.

[21] Thanga Selvi R., Muthulakshmi I. (2021). An optimal artificial neural network based big data application for heart disease diagnosis and classification model. *Journal of Ambient Intelligence and Humanized Computing*.

[22] Li Y., Yang Z., Han K. (2020). Research on the clustering algorithm of ocean big data based on self‐organizing neural network. *Computational Intelligence*.

[23] Tian B. (2019). Big data machine learning unde37r the framework of distributed computing. *Electronic Technology and Software Engineering*.

[24] Song H., Dai J., Zhang W. (2018). Partial discharge pattern recognition based on deep convolutional network under complex data sources. *High Voltage Technology*.

[25] QIAN F. (2019). Research on RBF neural network evaluation model of shipbuilding suppliers based on big data. *Ship Science and Technology*.

[26] Zhou L. (2018). Research on big data analysis method based on neural network algorithm. *Electronic Design Engineering*.

[27] Rubtsova N. B., Perov S. Y., Belaya O. V., Konshina T. A. (2020). New aspects of power grid facilities personnel workplaces electromagnetic environment. *Russian Journal of Occupational Health and Industrial Ecology*.

[28] Qu Y., Huang B., Han Y. (2019). Big data classification method based on improved neural network and ELM. *Information Recording Materials*.

[29] Lin Q.. (2019). Big data multi-label attribute classification technology in cloud service environment. *Microelectronics & Computer*.

[30] Lv C., Xing Y., Zhang J. (2017). Levenberg–Marquardt backpropagation training of multilayer neural networks for state estimation of a safety-critical cyber-physical system. *IEEE Transactions on Industrial Informatics*.

[31] Wei W., Ke Q., Nowak J., Korytkowski M., Scherer R., Woźniak M. (2020). Accurate and fast URL phishing detector: a convolutional neural network approach. *Computer Networks*.

[32] Yan Z., Chen J., Hu R., Huang T., Chen Y., Wen S. (2020). Training memristor-based multilayer neuromorphic networks with SGD, momentum and adaptive learning rates. *Neural Networks*.

[33] Tang S. (2019). Application of neural network technology based on big data in classroom face recognition. *Intelligent Computers and Applications*.

[34] Fekri-Ershad S. (2020). Bark texture classification using improved local ternary patterns and multilayer neural network. *Expert Systems with Applications*.

[35] Abbasi S. F., Ahmad J., Tahir A. (2020). EEG-Based neonatal sleep-wake classification using multilayer perceptron neural network. *IEEE Access*.

[36] Wang H., Zhao Y. (2019). Supplier selection of construction enterprises based on neural network in big data environment. *Journal of Civil Engineering and Management*.

[37] Theodoridis C. A., Kafka K. E., Perez A. M. (2016). Evaluation and testing of junctional tourniquets by special operation forces personnel: a comparison of the combat ready clamp and the junctional emergency treatment tool. *Journal of special operations medicine: A Peer Reviewed Journal for SOF Medical Professionals*.

[38] Fischer C., Pardos Z. A., Baker R. S. (2020). Mining big data in education: affordances and challenges. *Review of Research in Education*.

[39] Atat R., Liu L., Wu J., Li G., Ye C., Yang Y. (2018). Big data meet cyber-physical systems: a panoramic survey. *”IEEE Access*.

[40] Fang F. (2018). Research on big data analysis method based on neural network algorithm. *Software Engineering*.

[41] Zhang L., Zhang Y. (2016). Infinite depth neural network method for big data analysis. *Computer Research and Development*.

[42] Sun E. H. (2020). Social big data analysis based on recurrent neural network and fast text. *Computer Programming Skills and Maintenance*.

[43] Wu J., Guo S., Li J., Zeng D. (2016). Big data meet green challenges: big data toward green applications. *IEEE Systems Journal*.

[44] Zhou X., Hu Y., Liang W. (2020). Variational LSTM enhanced anomaly detection for industrial big data. *IEEE Transactions on Industrial Informatics*.

